RETRACTED

# An ML-Enabled Internet of Things Framework for Early Detection of Heart Disease

**DOI:** 10.1155/2022/3372296

**Published:** 2022-09-21

**Authors:** Yar Muhammad, Moteeb Almoteri, Hana Mujlid, Abdulrhman Alharbi, Fahad Alqurashi, Ashit Kumar Dutta, Sultan Almotairi, Hamad Almohamedh

**Affiliations:** ^1^School of Computer Science and Engineering, Beihang University, Beijing, China; ^2^Department of Management Information Systems, Business Administration College King Saud University, Riyadh 11451, Saudi Arabia; ^3^Department of Computer Engineering, Faculty of Computer Engineering, Taif University, Taif, Saudi Arabia; ^4^Computer Sciences and Information Department, Applied College, Taibah University, Al Madinah Al Munawwarah, Saudi Arabia; ^5^Department of Computer Science, Faculty of Computing and Information Technology, King Abdulaziz University, Jeddah 21589, Saudi Arabia; ^6^Department of Computer Science and Information Systems, College of Applied Sciences, Al Maarefa University, Riyadh 13713, Saudi Arabia; ^7^Department of Natural and Applied Sciences, Faculty of Community College, Majmaah University, Majmaah, 11952, Saudi Arabia; ^8^Department of Information Systems, Faculty of Computer and Information Sciences, Islamic University of Madinah, 42351, Saudi Arabia; ^9^Faculty of King Abdulaziz City for Science and Technology (KACST) Riyadh, Riyadh, Saudi Arabia

## Abstract

Healthcare occupies a central role in sustainable societies and has an undeniable impact on the well-being of individuals. However, over the years, various diseases have adversely affected the growth and sustainability of these societies. Among them, heart disease is escalating rapidly in both economically settled and undeveloped nations and leads to fatalities around the globe. To reduce the death ratio caused by this disease, there is a need for a framework to continuously monitor a patient's heart status, essentially doing early detection and prediction of heart disease. This paper proposes a scalable Machine Learning (ML) and Internet of Things-(IoT-) based three-layer architecture to store and process a large amount of clinical data continuously, which is needed for the early detection and monitoring of heart disease. Layer 1 of the proposed framework is used to collect data from IoT wearable/implanted smart sensor nodes, which includes various physiological measures that have significant impact on the deterioration of heart status. Layer 2 stores and processes the patient data on a local web server using various ML classification algorithms. Finally, Layer 3 is used to store the critical data of patients on the cloud. The doctor and other caregivers can access the patient health conditions via an android application, provide services to the patient, and inhibit him/her from further damage. Various performance evaluation measures such as accuracy, sensitivity, specificity, F1-measure, MCC-score, and ROC curve are used to check the efficiency of our proposed IoT-based heart disease prediction framework. It is anticipated that this system will assist the healthcare sector and the doctors in diagnosing heart patients in the initial phases.

RETRACTED

## 1. Introduction

Heart disease is a fatal illness that affects the heart and blood vessels. The common symptoms associated with this disease consist of squatness of inhalation, dimness of body, distended feet, obesity, stress, and tiredness with associated symptoms. [1]. One major cause of this disease is the life style of an individual. Smoking, high blood pressure, high cholesterol, a wholesome diet, obesity, and lack of exercise are the contributing factors for this disease [2]. Heart disease has various types, such as coronary heart disease (CAD), heart arrhythmia, failure, value, pericardial, cardiomyopathy (heart muscle disease), congenital (cardiac illness at birth), and cardiovascular heart disease (CVD). The most common type is CAD (narrowed or blocked coronary arteries), which causes chest discomfort, heart attack, and stroke. According to a report generated by WHO, in 2016, approximately 18 million people died from CVD, demonstrating 32.5% of total deaths worldwide. Among these deaths, 86% were due to stroke and heart failure. About 52–54% of the patients having this disease expires in the initial 1–2.5 years. The associated charge for the management of heart patients is around 4.1% of the yearly financial budget for healthcare [3]. Besides financial costs, heart disease greatly affect the economic and social status of a person, which indeed is very necessary for living a normal life.

CAD is amongst the most common cardiac diseases across the globe. In conventional approaches, angiography is deliberated as the most precise and common technique for identifying and detecting CAD. However, this approach has various drawbacks that degrade its significance. The conventional approaches used to detect and diagnose the cardiac disease are time-consuming and complex [4]. The treatment and diagnosis in under-developed countries are very complex because of the unavailability of medical diagnostic technology and expert physicians [5]. These conventional methods are based on the investigation of the patient's previous medical record, symptoms analyzed by the physicians, and mental and physical checkup reports. In addition, these approaches can cause inaccurate results due to human negligence. Further, considering the importance and damage caused by heart disease, it is necessary to identify and diagnose it in the initial phases [6].

RETRACTED

Nowadays, people are changing their living standards and are looking for ways to make their lives easier based on advanced technologies. The advancement in technologies has taken the world into a new era, in which all the basic needs of a human are not so far away. Advanced technologies and monitoring schemes play a significant part in everyday life like industries, control systems, agriculture, health, etc. Healthcare is the most prominent one, as it is very necessary for every human being. The advanced technologies have several applications in healthcare in which the Electronic Health Record (EHR) and control mechanism are very important [7]. The EHR offers a significant part in maintaining the clinical records of patients, which is very helpful in meeting the medical timelines. At the same time, the control mechanism assists in delivering the control strategies. The attachment or implanting of smart devices to/in the human body helps capture vital signs like BP, RR, EEG, ECG, sugar level, etc., of a patient in the smart healthcare system. Due to its characteristics and applications in healthcare, the IoT has attained an excessive devotion in the recent decades and is a go to approach for the researchers.

Traditionally, Structured Query Language- (SQL-) based databases were mainly used for storing the clinical data of patients. Nowadays, the IoT smart devices are increasing exponentially in quantity, quality, and variety, which monitor the patient's activities, fitness, and health status on a continuous basis. These wearable sensor devices produce an enormous volume of data which is not easy to store in conventional databases and data storage tools. Keeping this issue in mind, researchers have started using NoSQL (Non-Structured Query Language) and big data technologies in various IoT applications.

To tackle the problems associated with the early approaches, this paper proposes an efficient and scalable automated system that stores and processes a massive amount of heart-related data and monitors the real-time health condition of a patient. To increase the scalability and availability of the system, it is interconnected with cloud computing technologies. Our proposed health monitoring system is composed of three layers. At the first layer, IoT smart devices are attached to the body of the patients to collect different biological parameters. At the second layer, these collected parameters are processed using various ML classification algorithms. Finally, the third layer is used to store the critical data of a patient, which can then be accessed by physicians and other care-givers via an android application. The core contributions of this paper are given as follows:

- This study proposes a novel three-layer architecture based on ML and IoT technologies to monitor the health conditions of a patient with heart disease. IoT is used to capture those physiological parameters from the patient's body that have a strong impact on heart disease. The proposed healthcare framework is scalable and is based on advanced technologies that can store and process a massive amount of patients' critical clinical data in the cloud and also maintain the EHR of the patients
- The proposed framework is well-organized, energy-efficient, cost-effective, and offers low-latency services. The android app plays a key role in reducing latency, as the caregiver can access the health status of the patient with ease, with just a single click
- In the proposed framework, IoT devices are used to capture the important clinical measure and send it to the second layer. In the second layer, various ML classification algorithms are used for the accurate and efficient diagnosis of patients with heart disease at the early stages. This results in an automated model based on ML and IoT technologies, which is more scalable, cost-effective, and up to the mark
- In the proposed system, there is an automatic alert system as well, which alerts the doctor and other caregivers when the patient's health condition deteriorates
- The experimental and analysis results illustrate that the proposed system is much better than the earlier approaches/systems

The remaining article is structured as follows: Section 2 shows the related work, section 3 illustrates the material and methods, section 4 demonstrates our analytical model, while section 5 signifies the experimental outcomes. At last, in section 6 the whole paper is concluded.

RETRACTED

## 2. Related Work

Different ML classification algorithms like AdaBoost (AB), support vector machine (SVM), decision tree (DT), naïve Bayes (NB), logistic regression (LR), artificial neural network (ANN), etc. have been used extensively by different researchers for the identification and prediction of various diseases in healthcare. For example, Samuel et al. [8] used an ensemble technique for the analysis of cardiac illness and achieved an accuracy of 87.0%. Sundarasekar et al. [9] used a hybrid approach based on ANN and a fuzzy analytics hierarchy for the detection of cardiac disease and attained 88.3% of accuracy. Muhammad et al. [10] used a computational framework for the identification and detection of cardiac illness and conquered promising outcomes. All these approaches were applied to non-real-time data.

Keeping the damage caused by various diseases in mind, researchers have used IoT and AI techniques for observing the health disorders of a patient in a continuous manner. IoT is an interconnection of several physical objects used to perceive real-time events on continuous basis. These physical objects share data with each other with the help of wireless technologies and sensor nodes [11]. IoT-based systems follow a layered structural design for the transmission of data and signals among the connected devices. RFID tags, sensors nodes, and actuators are often used in IoT, and for mutual interaction between the connected IoT nodes unique addressing schemes are used [12].

Different researchers have used advanced technologies such as IoT, AI, fog computing, and big data in different fields for various purposes [13, 14]. For example, Ngabo et al. [15] proposed a recommendation system based on IoMT and ML for patient diet. Ishaq et al. [16] described various opportunities and applications of IoT in business organizations, discussing how IoT technologies are beneficial for business organizations. Harvard University developed a healthcare project named CodeBlue [17]. The main objectives of this project were to measure and monitor an individual's health parameters like EMG, ECG, and EKG. Alarm-Net was another project developed by the University of Virginia and the main objective of this project was to develop a framework that can monitor patient health on a continuous basis [18]. It uses the IP-based network for enabling wireless communication between networked devices [19, 20]. Blum and Magill [21] have developed a healthcare project named MobiCare that remotely determines the patient's health parameters. Their project measures the biological vitals parameters of a patient comprehensively and then forwards it to a doctor and other care providers through cloud computing technologies. To measure the mental health conditions of a person, Islam et al. [22] have developed another healthcare project named PAM.

Fog and cloud computing-based systems perform an important role in providing real-time and on-demand services to users over the Internet [23]. These systems have attracted researchers from various fields, e.g., academics, industrial partners, and healthcare professionals. Cloud computing has a major drawback though: it incurs excessive network delays, thus infeasible for systems and applications that require on-time and on-demand responses. Advanced technologies such as IoT, fog computing, edge computing, and big data have attracted a lot of attention and have been used for different applications and purposes [24], facilitating storage, processing, and communication. Fog computing has one main advantage over cloud computing: it is more suitable for those applications where response time is very important [25, 26]. He et al. [27] have developed a healthcare system to accumulate patient data. They used various sensors like ECG, temperature, and respiration rate sensors to gather different physiological parameters. The health data of patients are forwarded to the cloud where it is stored. Response time is the key drawback of their proposed scheme that reduces its effectiveness. Cheng et al. [28] have proposed an IoT-based healthcare framework that incorporates the IoT devices with the cloud platform for storing the health parameters of a patient in a continuous manner and minimizing the execution time of a given task.

RETRACTED

Saponara et al. [29] have developed an in-home health monitoring system for collecting various physiological parameters like BP, weight, ECG, etc. After collection, the collected parameters are sent to the hospital for monitoring the health status of a patient remotely. Ali et al. [30] have suggested another IoT-based smart healthcare framework for measuring and monitoring several important signals, such as BP, body temperature, and ECG. The physician and other caregivers can access to these values via a mobile application. However, this system is generic and does not take into account the concerns related to specific diseases. Akrivopoulos et al. [31] have presented an IoT and Software-Defined Networking- (SDN-) based E-Health system, which collects patients' data through a smartphone using their voices and decides their health status on the basis of their voices. This system is restricted to small amounts of data and operates locally. Sanghera et al. [32] developed a healthcare framework that uses ECG signals to detect heart abnormalities [33]. This system has certain limitations, such as low accuracy and excessive computation time, reducing its performance. Choi et al. [34] have presented another healthcare scheme based on IoMT that provides healthcare services named Autonomous Patrolling System, which uses an analytical hierarchical process for distributing the load and energy equally among all nodes. A cloud simulated environment is used for testing this system. The model performs well in terms of energy consumption but consumes more time when the nodes communicate with each other in order to process the requests of patients.

Mahmud et al. [35] proposed a healthcare scheme for predicting the probability of a cardiac attack. They compare their model with the RNN model, showing that their model works well on datasets of small sizes, but the performance and accuracy reduces on large data. Abdelmoneem et al. [36] have developed another system to overcome the latency problem associated with cloud computing approaches. Further, they measure the effectiveness of their system in terms of energy consumption and delay via the iFogSim simulator [37]. Sahoo et al. [38] suggested another model based on ML and fog computing, called FogLearn, for the identification and diagnosis of diabetes. Abdelmoneem et al. [36] developed an IoT and cloud computing-based system to measure the real-time health conditions of a patient. Further, a mechanism is proposed for the allocation of tasks among nodes, while the performance of this framework was evaluated through the iFogSim simulator [39].

RETRACTED

To solve the challenges associated with existing approaches, this study proposes a three-layer architecture based on IoT and ML technologies to monitor in real-time the health conditions of a patient with heart disease. Various ML classification algorithms are used for the accurate and efficient identification of patients with the cardiac disease at the early stages. Various challenges [40–46] that need to be solved to take advantage of the capacity of healthcare frameworks based on advanced technologies are as follows: (1) a scalable and effective advanced technology-based healthcare framework is needed that can process and store massive amounts of patient health data generated via sensor nodes, (2) a well-organized healthcare framework is required which is energy-efficient and offers low-latency services, and (3) the deployment of an automated ML model which can diagnose and detect the heart conditions accurately and effectively. We analyze our proposed prediction model and compare it with other existing models and approaches. The evaluation results demonstrated that the proposed system performs really well and outclass other models and approaches in terms of performance.

## 3. Material and Methods

The data used and the techniques followed for the accomplishment of this study are discussed in detail in this section. The following subsections elaborate on all the steps taken for the accomplishment of the proposed work.

### 3.1. Dataset

The primary and vital step of developing a smart system is to create or develop a dataset that is more related to the problem and that effectively and accurately imitates the target class patterns. A dataset that is more related to the problem and is well-organized improves the efficiency of the model. A Hungarian heart disease dataset has been utilized in this paper [46]. The dataset used is composed of 1025 instances in which 500 cases are positive while the rest are negative. The dataset consists of 13 features and a target label. The target label consists of two classes i.e. existence or nonexistence of cardiac disease.

RETRACTED

### 3.2. Preprocessing Techniques

The procedure of transforming raw data into understandable patterns is called data preprocessing. These techniques play a significant part in the representation of data in a well-organized and normalized form. Standard Scaler and Min-Max scaler are the two frequently used preprocessing techniques and are also used in this study in order to present the data to the classifiers and to increase the classification accuracy.

### 3.3. Proposed IoT and ML-Based Healthcare System

Our proposed healthcare framework consists of a three-layer architecture that stores and processes a large amount of healthcare data. Layer 1 collects data from wearable/implanted nodes. Layer 2 is used to process and store the data locally at the web server. Layer 3 is used to store such a large capacity of data collected at Layer 1 in the cloud.  Figure 1 explains the proposed system.

Figure 1 depicts the proposed IoT and ML-enabled framework for the early diagnosis of heart patients. Basically, Figure 1 consists of three layers in which Layer 1 is used to collect different physiological parameters like EEG, ECG, EMG, BP, etc., from the patient's body using different sensor nodes. Every physiological measure has its own threshold value, which indicates whether the value is normal or abnormal. After the collection of these measures, it sends the values to the second layer. The values are presented to the ML models, which decide whether the patient has heart disease or not. If the health conditions of the patient are not normal, it sends an alert message to the doctor. The doctor then prescribes the first aid and proper medication to the patient and helps him/her from further loss. After the classification in the second layer, the data is then forwarded to the third layer where it is stored. The third layer stores a large volume of patients' clinical data, and also maintains the EHR of patients. The doctor and other caregivers can access the EHR of the patients for future treatment. The layers of the proposed framework are discussed in detail.

#### 3.3.1. Layer 1

At the first layer of our proposed health monitoring system, IoT smart sensor nodes are implanted/fixed on an individual's body to accumulate various physiological measurements. These IoT nodes assemble data from the patient's body in a continuous manner. Every biological parameter has its own threshold rate. When it exceeds its standard rate, an alert message is sent to the practitioner and other caregivers along with its value. The collected data of a patient is then forwarded to a web server where it is stored and processed. Both the critical and normal values are stored in a continuous manner.  Figure 2 demonstrates an android-based data assistance interface of the proposed system.

RETRACTED

#### 3.3.2. Layer 2

This layer of the proposed framework is used for storing and processing the data on a web server and is called the data processing and storage layer. It collects the data from the first layer. After collecting the data, various preprocessing techniques like Min-Max and Standard Scaler are applied to it before presenting to the ML classifiers. The ML classifiers used include LR, MLP, RF, and SVM. Various performance metrics like accuracy, specificity, and sensitivity, etc., were used to track the efficiency of utilized ML models. After evaluating the biological data of a patient, the data is then forwarded to cloud storage in order to maintain the Electronic Health Record (EHR) of the patient, which is then accessed by physicians and other caregivers via an Android application.

#### 3.3.3. Layer 3

This layer of the proposed system is also known as the data storage or cloud layer. The data produced by the IoT smart devices are very large in volume, and is difficult to store in the conventional database technologies and tools. Physical devices and personal computers flop in storing such an enormous amount of data under such situations. To resolve this issue, this paper presents a scalable big data approach for storing such a large volume of clinical data in the cloud firebase, which is accessible from an Android Application when required by the doctor and other caregivers. To maintain the elasticity and scalability, the proposed system utilizes the cloud computing technology, i.e., Google Firebase. In order to create a real-time database which is used to store the real-time data coming from the second layer, firstly an account is created with the Google Firebase. Only the critical data of a patient will be stored here.  Figure 3 signifies the workflow of the proposed system.

From figure 3 we can observe that the wearable sensor nodes collect the biological measures from the patient's body and passes it to the healthcare holders such as a doctor. Based on the health conditions, the doctor prescribes proper medications and provides healthcare services. If the patients' health conditions deteriorate, the doctor provides emergency services and helps in saving their lives.

Figure 4 demonstrates the dataflow of the proposed healthcare system.

### 3.4. Performance Measuring Parameters

To measure the efficiency of various utilized ML models, different performance metrics are calculated. These measures are accuracy, sensitivity, specificity, etc. All these performance metrics can be measured from the confusion matrix as presented in Table 1.

RETRACTED

*True Negative (TN).* TN demonstrates that a person does not have the disease and the classifier also forecasts that he/she has no disease. It means that a healthy person is properly predicted by the classifier

*True Positive (TP).* TP shows that a person is a cardiac patient and the model also diagnoses him/her as a heart patient by doing a correct prediction

*False Positive (FP).* FP notifies that a person does not have heart disease, but the model does a wrong prediction by predicting him/her as a cardiac patient

*False Negative (FN).* FN represents that a person is cardiac patient, but the model does a wrong prediction by declaring him/her as a healthy person

*Accuracy.* Accuracy demonstrates the inclusive efficiency of algorithm, and it can be calculated via the following formula:

(1) $$\begin{array}{c} \text{Accuracy}=\frac{\text{TP}+\text{TN}}{\text{TP}+\text{FP}+\text{FN}+\text{TN}}*100\%\; \end{array}$$

*Specificity.* It is the ratio of the person classified as healthy by the model to the total number of healthy persons. This elaborates that the model predicted the individual as healthy. Its formula is given below:

(2) $$\begin{array}{c} \text{Specificity}=\frac{\text{TN}}{\text{TN}+\text{FP}}*100\% \end{array}$$

*Sensitivity.* It is the ratio of the person classified as a cardiac patient by the model to the total number of suspected patients. This shows that the model predicted a person as a heart patient. Its formula is given below:

(3) $$\begin{array}{c} \text{Sensitivity}=\frac{\text{TP}}{\text{TP}+\text{FN}}*100\% \end{array}$$

*F1-measure.* It is interpreted as the weighted average of the recall and precision. It has a value between 0 and 1, where 1 represents perfect value of F1 and shows good performance while 0 represents complete failure of the model and shows bad performance. The formula for F1-measure is:

(4) $$\begin{array}{c} \text{F}1\text{ score}=2*\frac{\text{precision}*\text{recall}}{\text{precision}+\text{recall}} \end{array}$$

*MCC.* It shows a correlation between the actual class and the class predicted by the model. Its value ranges between -1 and 1, where -1 demonstrates complete failure of the classification model while 1 shows the perfect and ideal prediction while 0 shows the random prediction of the model. Its formula is given below:

(5) $$\begin{array}{c} \text{MCC}=\frac{\text{TP}\times \text{TN}-\text{FP}\times \text{FN}}{\sqrt{\left(\text{TP}+\text{FP}\right)\left(\text{TP}+\text{FN}\right)\left(\text{TN}+\text{FP}\right)\left(\text{TN}+\text{FN}\right)}}*100\% \end{array}$$

At last, we examined the probability of the utilized ML classifiers using the ROC curve, which signifies the performance of classification models graphically.

RETRACTED

## 4. Analytical Model

### 4.1. Network Model

An undirected graph is used to represent our network model, *G* = [*V*, *E*, *W*], which includes a collection of IoT devices, a fog device, and a cloud server (*V* = *S*_*I*_ *U* *S*_*F*_ *U* *S*_*C*_). The ‘*E*' here represents a set of edges that shows the communication links among nodes. The ‘*W*' defines the collection of weights on edges. Here the tuple (*X*, *R*) is used to show the weights of edges, where *X* indicates the delay of propagation, while the *R* defines the communication degree between two devices. Besides the previously discussed logical three-layer architecture, we will not leave any topology constraints as this makes the presentation of the model easy.

### 4.2. Service Delay

Since the IoT devices are able to process the requests locally or send them to the fog node or cloud. The service delay of the IoT device ‘*i*' is signified by ‘*D*_*i*_'. The following formula is used to calculate it:

(6) $$\begin{array}{c} D_{i}=P_{i}^{I}.\left(Ai\right)+P_{i}^{F}.\left(X_{ij}^{\text{IF}}+Y_{ij}^{\text{IF}}+Lij\right)+P_{i}^{C}.\left(X_{ik}^{IC}+Y_{ik}^{IC}+Hk+X_{ki}^{CI}+Y_{ki}^{CI}\right), \end{array}$$

(7) $$\begin{array}{c} J=f\;\left(i\right),k=g\;\left(i\right). \end{array}$$

In the above equation, *P*_*i*_^*I*^ represents the likelihood of IoT node ‘*i*' to process its personal invitation at the first layer, where *P*_*i*_^*F*^ demonstrates the likelihood of the IoT node to forward its invitation to the fog layer, and *P*_*i*_^*C*^ is the likelihood of IoT node to send its request to the cloud layer directly. It may be noted that the summation of all probabilities is always equivalent to 1, i.e., *P*_*i*_^*I*^ + *P*_*i*_^*F*^ + *P*_*i*_^*C*^ = 1. *A*_*i*_ shows the mean delay of processing when the IoT node ‘*i*' processes its individual request.  *X*_*ij*_^IF^ represents the delay of the IoT node ‘*i*' to the fog nod ‘*j*', while *Y*_*ij*_^IF^ shows the total transmission delays from the IoT node ‘*i*' to the fog node ‘*j*'. Likewise, *X*_*ik*_^*IC*^ represents the delay of propagation from IoT node ‘*i*' to the cloud server ‘*k*', while the total sum of all the communication delays from IoT nodes to the cloud server is denoted by *Y*_*ik*_^*IC*^. Likewise, the transmission and propagation delays from the cloud server ‘*k*' to the IoT node ‘*i*' is denoted by *Y*_*ki*_^*CI*^ and *X*_*ki*_^*CI*^, respectively.

### 4.3. Delays in Fog Layer

Here in this subsection we have defined a recurrent equation for *L*_*ij*_, i.e., *L*_*ij*_ (*x*). This equation represents the processing delay and control the request of IoT node in the fog layer and probably the cloud as well, by the fog node *j* throughout the *X*^th^ offload in the fog layer (*x* ≥ 0). *P*_*j*_ represents the likelihood that the invitation is acknowledged by the fog node. The following equation is used to calculate L_ij_ (x):

(8) $$\begin{array}{c} Lij\;\left(x\right)=P_{j}.\left(Wj+X_{ji}^{FI}+Y_{ji}^{FI}+Lij\left(x+1\right)+\left(1-Pj\right)\right).\left[\left(1-O\left(x\right).\left(X_{j\text{ɉ}}^{FF}+Y_{j\text{ɉ}}^{FF}+Li\text{ɉ}\left(x+1\right)\right)\right)+O\left(x\right).\left(X_{jk}^{FC}+Y_{jk}^{FC}+Hk+X_{ki}^{CI}+Y_{ki}^{CI}\right)\right], \end{array}$$

where *W*_*j*_ demonstrates the mean wait time at the fog node, while *O*(*x*) represents the offload function. When the request of an IoT node ‘*i*' arrives at the fog layer, the fog node attempts to operate on the request first. The request is submitted to the processing queue and its probability is denoted by *P*_*j*_, when the request fails in entering to the processing queue its probability is (1 − *P*_*j*_), this is dependent on the expected waiting time. When the request arrives at queue, it shall encounter the mean waiting time *W*_*j*_, and the transmission and propagation delay of *Y*_*ji*_^*FI*^ and *X*_*ji*_^*FI*^, respectively, in order to go back to the IoT node.

RETRACTED

In case when the request does not enter to the fog node, then it will deposit the invitation to its finest neighbor at the fog layer denoted by *ɉ*, doing so will increase both the propagation and transmission delays, i.e., *X*_*jɉ*_^*FF*^ and *Y*_*jɉ*_^*FF*^, respectively. Further, this request also undergoes processing delay and controlling the request in the second layer, i.e., *L*_*iɉ*_ (*x* + 1). *X*_*jk*_^*FC*^ and *Y*_*jk*_^*FC*^ denote the transmission and propagation delay of the requests from fog layer to the cloud server. *H*_*k*_ denotes the cloud processing delay, while *X*_*ki*_^*CI*^ and *Y*_*ki*_^*CI*^ demonstrate the propagation and transmission delays, respectively.

## 5. Results and Discussion

The simulation outcomes achieved via different ML models used in this study are discussed here in this section. All the simulations are carried out using laptop systems having the following specifications. The specification of the system are as follows: model HP Elitebook G5, intel core i7, 9^th^ generation, having 16 GB RAM, and operates on Microsoft Windows 10. All the simulation results were conducted using Anaconda Jupyter Notebook as a simulation tool. Python has been used a language for the implementation purpose. The major packages used were Sklearn, Seaborn, Matplotlib, Pandas, Numpy, etc. To check the efficiency of each ML model, various performance metrics are computed.

RETRACTED

### 5.1. Performance of All Classification Algorithms

All the experiments and the experimental results achieved via various ML classifiers are represented in this section. The simulation results attained via the utilized classifiers are shown in Table 2.

Table 2 shows that KNN at “k =3” performed brilliantly and outclassed all the other models by achieving the accuracy of 96.09%, specificity of 95.99%, sensitivity of 96.19%, recall of 96.34%, 96.28% of precision, AUC of 99.09%, F1-score of 0.96, and 0.92 of MCC, and attained first position in terms of performance. RF attained the second spot in terms of performance, and achieved 95.70%, 96.19%, and 96.20% of accuracy, specificity, and sensitivity, respectively. The third best classifier was SVM (“kernel = rbf”). SVM (“kernel = rbf”) achieved 93.94% of accuracy, 94.18% of specificity, and 93.72% of sensitivity. The lowest performance was observed for NB classifier, i.e., accuracy of 82.33%, specificity of 78.15%, and sensitivity of 86.30%, and stood last in the performance competition.

Figure 5 illustrates the performance (accuracy, specificity, and sensitivity) of all classifiers utilized in this study.

From Figure 5 it is quite obvious that the KNN classification model outclasses all the other models in terms of the mentioned performance measures. RF also performed well and attained promising results in terms of the mentioned performance measures. NB showed bad performance and stood last in this regard.

Figure 6 notifies the recall, precision, and AUC of the investigated ML models. From Figure 6 it is apparent that KNN at “k =3” performed better than the other utilized classification models in terms of all these measures.

Again, in terms of precision, recall, and AUC scores, KNN left behind all the other models. Like the accuracy, sensitivity, and specificity, NB performed poorly and stood last in terms of precision, recall, and AUC scores.

Figure 7 represents the F1 and MCC scores of all the utilized classifiers. Once again KNN at “k =3” outclassed the rest of the classifiers in terms of F1 and MCC-score.  Figure 8 demonstrates the ROC curves of different models used in this paper.

Multiple experiments were performed for various values of ‘*K*'.  Table 3 demonstrates the simulation results of the KNN classifier accomplished via multiple experiments for different values of *K*, i.e., from “k=3 to 10”.

Table 3 describes the results of the KNN algorithm on different K values (*k* = 3 to 10). The simulation outcomes show that at ‘*K* = 3' it shows superior performance and attained 96.09% accuracy.  Figure 9 graphically shows the performance of the KNN model by conducting multiple experiments.

RETRACTED

Table 4 illustrates the statistical analysis such as chi-square and *p*-value of the investigated models.

Furthermore, we conducted a comparative study of our work with the existing state-of-the-art approaches as mentioned in the literature review. The classification accuracies of the earlier approaches is illustrated in Table 5. From Table 5 it is quite obvious that the proposed system is way better in terms of accuracy and other evaluation metrics as compared to the earlier methods.

## 6. Conclusion

Heart disease is a hazardous and lethal disease which is growing at a faster speed all over the world and increasing the death ratio. Heart disease normally occurs due to the failure of the heart in supplying a sufficient volume of blood to supplementary parts of the body. Early and on-time diagnosis of cardiac disease can significantly reduce the damage caused by this disease by providing proper treatment and medicines to the patients. Heart disease diagnosis and treatment in undeveloped countries is a difficult and complex process due to the scarcity of medical diagnostic tools, lacking specialist doctors, and other means which play a major role in the diagnosis and treatment of such disease. Various methods have been used for the diagnosis of cardiac disease, among which angiography is considered to be the most prominent one. But some major limitations are associated with this approach; for instance, the high cost which reduces the effectiveness of angiography. We proposed a scalable IoT and ML-based health monitoring framework for the early detection and identification of cardiac patients. The architecture of our proposed system consists of three layers. Layer 1 is used to collect various physiological parameters from a patient using sensor devices. Layer 2 stores and processes the data (applying ML classifiers) locally at a local web server. Numerous performance measures are used to track the efficiency of ML algorithms. Layer 3 is used to store the critical data of a patient at the cloud firebase, which can be accessed by both the practitioner and other caregivers through a mobile application. Layer 3 also stores and maintains the EHR of patients, which can then be used for further treatment in future. It is projected that this system will assist the caregivers in providing early and on-time services to the patient, and will help them in saving the patients' lives. The future work of this study is to use some security tools and algorithms that help in the protection of the patient's critical clinical data. The use of more vital techniques that help in the reduction of the processing delay is also one of the future work.

RETRACTED

## Figures and Tables

**Figure 1:** Proposed IoT and ML based Architecture.

**Figure 2:** Data assistant interface of Layer 1.

**Figure 3:** Workflow of the IoT and ML-based healthcare framework.

**Figure 4:** Dataflow diagram of the proposed IoT and ML-based healthcare framework.

**Figure 5:** Accuracy, sensitivity, and specificity results of all classifiers.

**Figure 6:** Precision, recall, and AUC results of all classifiers.

**Figure 7:** F1 and MCC-score results of all classifiers.

**Figure 8:** ROC curve results of all classifiers.

**Figure 9:** Performance of KNN at K (*K* = 3 to 10).

**Table 1:** Confusion Matrix.

	Predicted (-)	Predicted (+)
Actual (-)	TN	FP
Actual (+)	FN	TP

**Table 2:** Performance of all classification models.

Classifier	Accuracy	Specificity	Sensitivity	Recall	Precision	AUC	F1	MCC
MLP	84.96	80.76	88.97	88.99	83.02	91.79	0.86	0.70
LR (*C* = 1)	84.77	78.75	90.49	90.62	81.90	92.32	0.85	0.70
KNN (*K* = 3)	96.09	95.99	96.19	96.34	96.28	99.09	0.96	0.92
DT	86.82	83.76	89.73	89.89	85.40	91.89	0.87	0.74
AB	92.09	92.38	91.82	91.89	92.84	97.92	0.92	0.84
RF	95.70	96.19	96.20	96.24	95.20	99.28	0.96	0.92
SVM (kernel = linear, *C* = 1, gamma = 0.005)	84.19	75.95	92.01	92.09	80.27	91.46	0.86	0.69
SVM (kernel = rbf, *C* = 1, gamma = 0.005)	93.94	94.18	93.72	93.79	94.59	97.96	0.94	0.88
NB (Gaussian)	82.33	78.15	86.30	86.49	80.98	90.70	0.84	0.65

**Table 3:** Performance of KNN classification model at *K* (*k* = 3 to10).

KNN (model)	Accuracy	Sensitivity	Specificity
*K* = 3	96.09	96.19	96.09
*K* = 4	85.16	74.90	95.99
*K* = 5	76.87	75.09	78.75
*K* = 6	78.73	70.34	87.57
*K* = 7	75.70	76.99	74.34
*K* = 8	74.92	73.38	76.55
*K* = 9	78.14	80.98	75.15
*K* = 10	76.67	74.14	79.35

**Table 4:** Chi-square and p-value of all the classification models.

Classification model	Chi-square value	*p*-value (significance at *p* < .05)
MLP	149.6790	<0.00001
DT	196.9749	<0.00001
KNN (*K* = 3)	222.0388	<0.00001
DT	155.5049	<0.00001
AB	209.8046	<0.00001
RF	216.2733	<0.00001
SVM (linear)	143.9837	<0.00001
SVM (RBF)	190.1793	<0.00001
NB	133.2140	<0.00001

**Table 5:** Comparison of different research studies.

Research work	Method	Accuracy
Reference [47]	Hybrid system framework	87.05
Reference [48]	HRFLM	88.82
Reference [49]	Three-tier IoT architecture	89.98
Reference [50]	HealthFog	90.94
Reference [51]	Stacked SVM approach	92.32
Reference [10]	Intelligent computational framework	94.41
Proposed system	ML-enabled IoT framework	96.09

## Data Availability

All the data is available in the paper.
